RETRACTED

# Clinical Effect of Mudan Granule on Peripheral Neuritis Caused by Chronic Renal Insufficiency

**DOI:** 10.1155/2022/1052744

**Published:** 2022-03-31

**Authors:** Xinle Li, Huan Zheng, Zhihong Zhou, Zhao Li, Xiurong Zhou, Ming Zheng

**Affiliations:** Department of Neurology, Wuhan Wuchang Hospital (Wuchang Hospital Affiliated to Wuhan University of Science and Technology), Wuhan City, Hubei Province 430063, China

## Abstract

**Objective:**

To investigate the clinical effect of Mudan granule on peripheral neuritis caused by chronic renal insufficiency (CRI).

**Methods:**

Sixty patients with peripheral neuritis caused by CRI treated in our hospital were included from February 2018 to April 2021 in this study. The patients were arbitrarily assigned into control group and study group. The former accepted routine treatment, while the latter accepted Mudan granule treatment. The clinical efficacy, traditional Chinese medicine (TCM) clinical symptom score, nerve conduction velocity, hemorheology index, renal function index, and inflammatory factor index were compared.

**Results:**

We firstly compared the clinical efficacy: the study group was clinically cured in 22 cases, obviously effective in 5 cases, effective in 3 cases, and ineffective in 1 case, with a total effective rate of 96.67%. The control group was clinically cured in 9 cases, obviously effective in 8 cases, effective in 7 cases, and ineffective in 6 cases, with a total effective rate of 80.00%. The total effective rate of the study group was higher compared to the control group (*P* < 0.05). Secondly, we compared the TCM clinical symptom scores; before treatment, there exhibited no significant difference (*P* > 0.05); after treatment, the TCM clinical symptom scores decreased. The clinical symptom score of TCM in the study group was lower compared to the control group (*P* < 0.05). Compared with the control group, the nerve conduction velocity of left MCV, right MCV, left SCV, and right SCV in the study group were remarkably higher. In terms of the hemorheological indexes, the high-shear whole blood viscosity, low-shear whole blood viscosity, and plasma viscosity in the study group were lower compared with the control group (*P* < 0.05). Before treatment, there existed no significant difference in renal function indexes, but after treatment, the renal function indexes decreased, and the levels of serum creatinine (SCr), blood urea nitrogen (BUN), and uric acid (UA) in the study group were lower compared to the control group (*P* < 0.05). Finally, we compared the indexes of inflammatory factors; there existed no significant difference before treatment, but after treatment, the indexes of inflammatory factors decreased in both groups, and the levels of IL-6 and CRP in the study group were lower compared to the control group (*P* < 0.05).

RETRACTED

**Conclusion:**

For peripheral neuritis caused by CRI, Mudan granule can remarkably promote the clinical symptoms of TCM and reduce the syndrome score of TCM; moreover, it can remarkably increase the nerve conduction velocity of median nerve and common peroneal nerve and reduce blood viscosity, which is worth popularizing and developing in clinic.

## 1. Introduction

Chronic renal insufficiency (CRI) has become a global disease that needs to be paid more attention to [1]. The causes of CRI mainly include a variety of primary and secondary glomerular diseases, renal tubulointerstitial lesions, renal vascular lesions, and genetic factors, which act for a long time and show chronic onset, resulting in irreversible damage to nephron and renal function [1]. Its clinical manifestations are often water and electrolyte metabolism disorders, protein, carbohydrate, fat, and vitamin metabolism disorders and then affect the functional imbalance of multiple organs and systems. On February 20, 2007, the International Society of Nephrology issued a notice indicating that more than 500 million people worldwide have kidney diseases, which means that on average, one in ten people may suffer from kidney disease. Kidney disease can cause cardiovascular disease, and more than 1 million people die every year [2]. With the increasing number of patients with CRI, how to treat CRI better has become an urgent issue to be dealt with. With the continuous development of the disease, the renal metabolic function of patients with CRI is impaired, which will greatly increase the risk of peripheral neuritis when taking drug treatment [2, 3]. Peripheral neuritis caused by CRI is mainly caused by the disturbance of peripheral blood circulation. Patients often have limb numbness, dullness, or loss and pain as the main clinical manifestations, if intervention measures are not taken in time, severe patients may even face amputation, which has a great impact on their quality of life. At present, the pathogenesis of peripheral neuritis caused by CRI is not completely clear. Western medicine mostly believes that it is related to oxidative stress, abnormal activation of polyol metabolic pathway, endoplasmic reticulum stress, increase of advanced glycation end products, Na+/K+-ATP enzyme dysfunction, mitochondrial damage, inflammatory response, nerve growth factor deficiency, neuronal and glial cell apoptosis, and so on. Clinically, there is no radical cure mainly to improve metabolic disorders, supplemented by analgesia and nutritional nerve drugs, and the long-term effect is not ideal [3]. Therefore, doctors advocate to give full play to the advantages of TCM and actively explore the use of TCM or the combination of traditional Chinese and western medicine to treat the disease, in order to improve the clinical efficacy and reduce adverse reactions.

RETRACTED

Taking deficiency of both qi and yin and blood stasis ratio blocking collaterals as the pathogenesis, Mudan granule has been developed for many years which has become a commonly used clinical drug for the treatment of peripheral neuropathy and has the effects of replenishing qi and stagnation, enhancing blood circulation, relieving pain, and relieving blood stasis [4]. According to TCM theory, the remedy uses *Astragalus membranaceus*, which tonifies Qi and unblocks the blood vessels, supplemented by Chicken Blood Vine to move Qi and relieve pain, and *Panax ginseng* to invigorate blood and remove blood stasis to dispel pain. In addition, Radix Salviae Miltiorrhizae, Radix Paeoniae Rubra, and *Ligusticum chuanxiong* were employed to facilitate blood circulation and remove blood stasis. Modern pharmacology has found that *Astragalus membranaceus* can inhibit inflammatory factors and correct microcirculation. *Salvia miltiorrhiza* can correct blood flow, protect erythrocyte membrane from damage, inhibit the formation of atherosclerosis, and improve blood lipids. Rhizoma Corydalis has a significant effect on promoting blood circulation, relieving blood stasis, and relieving pain and has a high tolerance to hypoxia [5]. As an extract of *Ligusticum chuanxiong*, alkaloid ligustrazine can not only repair cerebral vessels and prevent and cure thrombosis, but also alleviate the performance caused by vitamin E deficiency [6]. Meta-analysis indicated that Mudan granule had a clear effect on diabetic peripheral neuropathy. It has a significant regulatory effect on diabetes with carotid arteriosclerosis, early diabetic nephropathy, diabetic autonomic neuropathy, and so on. However, at present, the application of Mudan granule in the treatment of peripheral neuritis caused by CRI is still lack of evidence-based basis. Based on this, the study focuses on the clinical efficacy of Mudan granule in the treatment of peripheral neuritis caused by CRI.

## 2. Patients and Methods

### 2.1. Clinical Information

Sixty patients with peripheral neuritis caused by CRI treated in our hospital were enrolled from February 2018 to April 2021. The patients were arbitrarily assigned into control group and study group. The former accepted routine treatment while the latter accepted Mudan granule treatment. In the control group, the age was 34-74 years old, with an average of 50.39 ± 3.65 years, containing 18 males and 12 females, while in the study group, the age was 35-76 years old, with an average of 50.43 ± 3.12 years, containing 16 males and 14 females. There exhibited no statistical significance in the general data. This study was permitted by the Medical Ethics Association of our hospital, and all patients noticed informed consent.

RETRACTED

Inclusion criteria are as follows: (1) age ≥ 18 years old and (2) in terms of the diagnostic criteria of peripheral neuritis caused by CRI in TCM and western medicine [7].

Exclusion criteria are as follows: (1) neuropathy caused by other causes, containing cervical and lumbar vertebra disease, cerebral infarction, severe arteriovenous vascular disease, and neurotoxicity caused by drugs and chemicals; (2) severe cardiac, liver and renal dysfunction [8]; (3) patients with malignant tumors; (4) those who cannot cooperate with clinical trials (patients with incomplete data); (5) those with increased complexity after comprehensive evaluation, such as unstable living environment and frequent changes in working environment; (6) patients with mental illness; (7) those who participated in clinical trials of other drugs in recent 1 month; and (8) those who had a history of alcoholism, psychotropic drugs, and drug dependence in the past 3 years.

Withdrawal criteria are as follows: (1) voluntarily withdrew from the trial; (2) poor compliance seriously affected the efficacy of the observation; (3) complicated with other serious lesions affecting the test results; (4) serious adverse reactions should not continue to receive treatment; and (5) courses of treatment did not end loss of follow-up or death of patients.

Shedding criteria are as follows: (1) those who fail to complete the course of treatment or drop out and (2) treatment of shedding cases: contact the patients actively, understand the reasons, make corresponding records, and keep files.

### 2.2. Treatment Methods

Control group: Mecobalamin tablets (manufacturer: Eisai (China) Pharmaceutical Co., Ltd.; approval no.: National Medicine H20143107; specification: 0.5 mg∗20 tablets) 0.5 mg po, tid; combined with iPASTER (Tanglin) tablets (manufacturer: Yangzijiang Pharmaceutical Group Nanjing Hailing Pharmaceutical Co., Ltd.; approval no.: Chinese Medicine H20040012; specifications: 50 mg∗10 tablets) 50 mg, po, tid.

The study group: Mudan granule (Huangqi 30 g, Rhizoma Corydalis 10 g, Sanqi 3 g, Radix Paeoniae Rubra 10 g, *Salvia miltiorrhiza* 10 g, Chuandongdong 6g, safflower 6 g, sappan 10 g, Jixueteng 30 g) (manufacturer: Liaoning Aoda Pharmaceutical Co., Ltd..) po, tid, combined with mecobalamin tablets 0.5 mg po, tid, and iPASTER (Tang Lin) 50 mg po, tid. (the manufacturers, approval numbers, and specifications of methyltyramine capsule and iPASTER tablets are the same as those in the control group). The patients were treated for 4 weeks as a course of treatment, with a total of 4 courses of treatment.

RETRACTED

### 2.3. Observation Index

#### 2.3.1. Curative Effect Evaluation

We judged the efficacy of TCM according to the 2002 edition of the Guidelines for Clinical Research on New TCM Drugs issued by the Ministry of Health of the People's Republic of China. The details are as follows: (1) clinical healing (the clinical symptoms and signs of TCM disappear or basically disappear); (2) significant reduction of clinical symptoms and signs of TCM and a 70% reduction in symptom score; (3) effective (clinical symptoms and signs of TCM improve and a 30% reduction in symptom score); and (4) ineffective (clinical symptoms and signs of TCM are not significantly promoted or even worsen and a 30% or less reduction in symptom score).

Note that the calculation formula (nimodipine method) is [(pretreatment integral − posttreatment integral)/pretreatment integral]∗100%.

#### 2.3.2. Clinical Symptom Score of TCM

The TCM clinical symptom scores of the patients before and after treatment were evaluated, respectively, and the TCM symptom grading quantitative table was employed to evaluate the main symptoms of limb numbness, limb pain, and abnormal temperature sensation, and in terms of the severity of the symptoms, the scores from mild to severe were 0, 2, 4, and 6, respectively, and the total score was 0-18.

#### 2.3.3. Nerve Conduction Velocity

The motor nerve conduction velocity (MCV) and sensory nerve conduction velocity (SCV) of bilateral median nerve, MCV of common peroneal nerve, and SCV of sural nerve were measured.

#### 2.3.4. Hemorheological Index

Fasting venous blood was taken to determine the hemorheological indexes: low-shear whole blood viscosity, high-shear whole blood viscosity, and plasma viscosity.

#### 2.3.5. Laboratory Index

Laboratory indexes such as serum creatinine (SCr), blood urea nitrogen (BUN), uric acid (UA), interleukin-6 (IL-6), and C-reactive protein (CRP) were analyzed.

### 2.4. Statistical Analysis

SPSS 21.0 statistical software was employed for data analysis, and *t*-test was employed for measurement data in accordance with normal distribution, expressed by $\bar{x}\pm s$, nonparametric test was employed for nonnormal distribution, and *χ*^2^ test was employed for counting data. The test standard *P* employs the bilateral test method, *P* < 0.05 indicates that there exhibited a significant difference in the statistical data, and *P* < 0.01 indicates that there exhibited a very significant difference in the statistical data.

RETRACTED

## 3. Results

### 3.1. Comparison of Clinical Efficacy

First of all, we compared the clinical efficacy: the study group was clinically cured in 22 cases, obviously effective in 5 cases, effective in 3 cases, and ineffective in 1 case, with a total effective rate of 96.67%. The control group was clinically cured in 9 cases, obviously effective in 8 cases, effective in 7 cases, and ineffective in 6 cases, with a total effective rate of 80.00%. The total effective rate of the study group was higher compared to the control group (*P* < 0.05). All the data results are indicated in Table 1.

### 3.2. Comparison of Clinical Symptom Scores of TCM

Secondly, we compared the TCM clinical symptom scores. Before treatment, there exhibited no significant difference (*P* > 0.05). The TCM clinical symptom score of the study group was lower compared to the control group (*P* < 0.05). All the data results are indicated in Table 2.

### 3.3. Comparison of Nerve Conduction Velocity

Thirdly, we compared the nerve conduction velocity. The left MCV, right MCV, left SCV, and right SCV in the study group were remarkably higher compared to the control group (*P* < 0.05). All the data results are indicated in Figure 1.

### 3.4. Comparison of Hemorheological Indexes

Then we compared the hemorheological indexes. The low shear whole blood viscosity, high shear whole blood viscosity, and plasma viscosity in the study group were lower compared to the control group (*P* < 0.05). All the data results are indicated in Figure 2.

### 3.5. Comparison of Renal Function Indexes

Next, we compared the renal function indexes; there exhibited no significant difference before treatment, but after treatment, the renal function indexes decreased, and the levels of SCr, BUN, and UA in the study group were lower compared to the control group (*P* < 0.05). All the data results are indicated in Table 3.

### 3.6. Comparison of Inflammatory Factor Indexes

Finally, we compared the indexes of inflammatory factors; there exhibited no significant difference before treatment, but after treatment, the indexes of inflammatory factors decreased, and the levels of IL-6 and CRP in the study group were lower compared to the control group (*P* < 0.05). All the data results are indicated in Table 4.

## 4. Discussion

With the increasing number of patients with CRI, CRI has become an important public health problem in the twenty-first century [9]. The epidemiological survey of CRI in China indicates that the prevalence rate of CRI in adults over 20 years old is about 10% [10]. There are many aspects of research and progress in the pathogenesis of CRI. These include glomerular hemodynamic changes: high filtration, high perfusion, and high transmembrane pressure in the glomerulus due to a variety of reasons. Under this high load, the nephron is constantly damaged, and renal function deteriorates and eventually enters end-stage renal disease [11, 12]. The damage of renal tubule and its interstitium is also an important factor in the progression of CRI, which is related to the high metabolism of renal tubules and the increase of oxygen consumption, which leads to the increase of oxygen free radicals, which leads to the formation of membrane attack complex and the activation of complement bypass [13]. Other studies have indicated that intestinal flora can also affect the progression of CRI [14]. The decline of renal function is irreversible, and the continuous decline of renal function index is the inevitable outcome of CRI. Clinically, whether it is to choose long-term hemodialysis, abdominal dialysis, or even kidney transplant treatment, the cost is still high; for most families, it is an unbearable economic burden. However, peripheral neuritis caused by CRI will not only increase the difficulty of disease treatment, but also increase the economic burden. Therefore, it is particularly important to delay the further deterioration of renal function and improve peripheral nerve function. It is particularly important to explore more effective and relatively cheap methods for the treatment of peripheral neuritis caused by CRI [15].

RETRACTED

Mudan granule is the first Chinese medicine preparation independently developed in China to treat peripheral neuritis. It is composed of Radix Astragali, Rhizoma Corydalis, *Panax notoginseng*, Radix Paeoniae Rubra, Radix Salviae Miltiorrhizae, *Ligusticum chuanxiong*, safflower, sappan wood, and chicken blood vine. In the prescription, *Astragalus* is sweet, lukewarm, and good at entering the spleen and stomach, which can not only replenish qi and blood, but also invigorate qi and blood, dispel blood stasis, and remove blood stasis. Chuanxiong Xin Tong, a “qi medicine in blood”, can pass through the whole body qi and blood, and its compatibility with *Astragalus* can enhance the use of facilitating blood circulation and relieving blood stasis and relieving pain. Both *Panax notoginseng* and Rhizoma Corydalis have the function of enhancing blood circulation. *Panax notoginseng* can not only activate blood circulation and relieve pain, but remove blood stasis. In the meantime, it also has the function of promoting qi circulation, qi stagnation in blood circulation, blood stagnation in qi, good treatment of pain up and down the body, combination of two drugs to enhance the effect of promoting qi, activating blood circulation and relieving pain, promoting qi circulation, dredging menstruation, and relieving pain. Radix Paeoniae Rubra and Radix Salviae Miltiorrhizae are bitter; mild cold has the effect of enhancing blood circulation, good blood circulation, and relieving blood stasis and relieving pain and is widely adopted in various blood stasis diseases; Honghua Xin San Wentong is compatible with Radix Paeoniae Rubra and *Salvia miltiorrhiza* which has the effect of facilitating blood circulation to enhance the power of enhancing blood circulation and relieving blood stasis; Su Mu Ganxian is good at entering the blood, mainly breaking blood, and good at enhancing blood circulation and relieving blood stasis and menstruation and relieving pain [15]. Chicken blood vine is gentle in nature and good at promoting blood circulation, invigorating blood, relaxing muscles, activating collaterals, and relieving blood stasis without harming. It is a common medicine for the treatment of obstruction of meridians and discord of collaterals caused by blood stasis. The combination of various medicines has the effect of tonifying qi and nourishing blood, relieving blood stasis, and relieving pain [16, 17].

RETRACTED

*Astragalus membranaceus* is an important medicine for tonifying middle and replenishing qi, which can not only tonify spleen, but also replenish blood and promote the formation and distribution of body fluid [18]. It is good at treating spleen deficiency and relieving thirst of body fluid. Entering the lungs can also replenish lung qi, which can be adopted for those with weak lung qi, shortness of breath, and mental exhaustion. It is good at invigorating qi and rising yang and is often adopted to treat the syndrome of depression of spleen deficiency and depression of qi in the absence of rising spleen yang. It can also be adopted to strengthen the surface and treat the syndrome of surface deficiency and spontaneous sweating. “Materia Medica Huiyan”: “tonifying the lung and invigorating the spleen, relieving sweat, expelling wind, and transporting drugs.” “The heart of medicine is recorded in the West”: “it can replenish qi, raise qi in the meantime, and be good at treating the depression of the atmosphere in the chest (that is, Zongqi).” Modern pharmacological studies have indicated that *Astragalus membranaceus* contains glycosides, polysaccharides, flavonoids, amino acids, and trace elements, which can promote body metabolism, improve anemia, increase hypoglycemia, reduce hyperglycemia, protect cardiovascular system, and reduce platelet adhesion. Astragalosides participate in biological processes such as energy supply, oxygen supply, protein, sugar, and fat metabolism [18, 19] and increase the activity of Na+/K+-ATP enzyme in nerve cell membrane. Protect P cells from hyperglycemia through strong antioxidation [19].

RETRACTED

Yanhusuoxin powder is good at treating the syndrome of qi and blood stasis and relieving pain. It is a good medicine for enhancing blood circulation and relieving pain. No matter what kind of pain, it can be adopted in combination with safflower, *Ligusticum chuanxiong*, and other blood-activating drugs to treat the pain of qi stagnation and blood stasis. “Lei Gong's Theory of Artillery”: “heartache to death, quickly looking for Yanhu.” Compendium of Materia Medica: “Rhizoma Corydalis, can carry out qi stagnation in blood, blood stagnation in qi, so it specializes in treating all kinds of pain up and down the body, which is wonderful in use. Gaiyanhusuo activating blood circulation and transforming gas, the first medicine is also.” Rhizoma Corydalis contains more than 20 kinds of alkaloids, among which tetrahydropalmatine has significant analgesic and sedative effects. The total alkaloids can dilate the peripheral blood vessels, activate blood circulation and benefit qi, increase blood flow, and improve hypoxia tolerance [20]. Studies have indicated that the analgesic effect of Rhizoma Corydalis is better compared to compound aspirin; its analgesic potency is 40% of that of morphine, and there is no addiction [21].

Panax notoginseng enters the liver meridian blood, is good at stopping bleeding, and can remove blood stasis and give birth to new. It can be adopted for all kinds of bleeding inside and outside the human body, no matter whether there is stasis or not, and it can activate blood circulation to resolve fatigue and pain, and it is often compatible in promoting blood circulation and qi medicine to enhance its power of promoting blood circulation and relieving pain. It is often adopted to treat injuries caused by falls or fractures of tendons, and it is an important medicine in the Department of Traumatology. In the meantime, this product also has the effect of tonifying deficiency, and it is often adopted to treat all kinds of deficiency injury. “Materia Medica seeking Truth”: “Panax notoginseng, the world only knows the function of stopping bleeding and stopping pain, but they do not know that pain is caused by blood stasis, and blood is stopped because of blood stasis. Panax notoginseng smells bitter and warm, and can differentiate its blood stasis in blood.”*Panax notoginseng* mainly contains saponins, and its main component of hemostasis is *Panax notoginseng*, which can resist platelet aggregation, promote the increment of hematopoietic stem cells, reduce myocardial oxygen consumption, promote body immunity, and has the effects of analgesia, anti-inflammation, and antiaging. Panax notoginseng saponins have significant hypoglycemic and slimming effects, effectively inhibit the activation of oxidase, inhibit oxygen free radicals, stress against antioxidation, and inhibit the activity of cysteine protease-3A. Thus, it can induce the expression of heat shock protein 70, inhibit apoptosis, restore protein kinase-B signal pathway, remarkably strengthen endothelial function, restrain aggregation and platelet adhesion, accelerate blood flow, and reduce blood viscosity. It can remarkably prevent and treat atherosclerosis [22, 23].

RETRACTED

Red peony is bitter cold and enters the liver meridian to invigorate the blood, good at clearing liver fire, Huo Xue Shan fatigue and pain, often used in treating blood fever and vomiting blood, red eyes and swelling pain, liver depression and downward pain, bruises, and injuries. It can remove the old blood and refresh the new blood [24]. Radix Paeoniae Rubra contains paeoniflorin and gallic tannic acid, which can inhibit platelet aggregation, and its decoction can prolong the time of thrombosis in vitro and reduce the dry weight of thrombus. Paeoniflorin can protect nerve cells by inhibiting apoptosis, activating adenosine receptor, blocking sodium channel, and reducing calcium overload injury. Paeoniflorin also has sedative, anti-inflammatory, and analgesic effects. Some studies have indicated that the antithrombotic effect of Radix Paeoniae Rubra is produced by inhibiting thrombin and activating plasminogen. It also has significant effects of reducing blood lipids and antiatherosclerosis, can remarkably improve the function of cardiovascular system, reduce the activity of reduced coenzyme II, and thus reduce oxidative stress [25].

*Salvia miltiorrhiza* is bitter in taste, good in enhancing blood circulation and relieving blood stasis, which can facilitate blood circulation and nourish blood [26]. It is widely adopted in all kinds of blood stasis diseases, especially in the treatment of blood stasis caused by blood heat and stagnation. The Compendium of Materia Medica: “it can break the old blood and replenish the new blood.” It is often employed to treat symptoms such as irregular menstruation, amenorrhea, postpartum blood stasis, and abdominal pain. *Salvia miltiorrhiza* mainly contains fat-soluble and water-soluble components, containing tanshinone, tanshinol, tanshinaldehyde, etc., which can improve microcirculation, inhibit the decrease of vascular endothelial cells caused by H202, reduce injury, protect vascular endothelium, promote blood flow, dilate blood vessels, improve hemorheology, reduce blood viscosity, and improve cell electrophoresis time and hematocrit in blood [26, 27]. Modern pharmacological studies indicate that *Salvia miltiorrhiza* can obviously inhibit a variety of coagulation factors, activate plasminogen activator, accelerate fibrinolysis, activate blood circulation, and relieve blood stasis and have sedative and analgesic effects on the central nervous system. It can also inhibit *Staphylococcus aureus*, *Leptospira*, bacilli, etc. [27].

RETRACTED

Ligusticum chuanxiong can reach the whole body qi and blood, which is the “qi medicine in the blood” [28]. It is good for regulating menstrual water and opening depression knot and is often adopted with red peony and peach kernel. It can treat a variety of gynecological diseases and is an important medicine for gynecology. Rhizoma Chuanxiong is known to regulate menstrual flow and open stagnant knots and is often employed together with Radix Paeoniae Alba and Peach Kernel. It can treat various gynecological diseases and is an important medicine in gynecology. It is pungent and warming, dispersing wind, relieving pain, and rising and inducing to treat headaches, as Li Dong Yuan once said "Chuanxiong must be used for headaches" and can be used in conjunction with any wind-cold, wind-heat, or rheumatic headache. Modern pharmacological studies have shown that Chuanxiong mainly contains alkaloids, volatile oils, and phenolic substances, of which Ligusticum can regulate Ca2+, inhibit Ca2+ influx, promote intracellular Ca2+ release, dilate coronary arteries, improve myocardial blood supply and improve microcirculation, inhibit platelet aggregation, and reduce platelet surface activity. Rhizoma Chuanxiong also inhibits excitation of the central nervous system and has sedative and hypnotic effects, as well as antihistamine and choleretic effects [28].

Safflower Xin San Wentong is an important medicine for facilitating blood circulation and relieving blood stasis and dysmenorrhea and reducing pain. It can activate blood circulation to relieve menstruation and relieve pain and can treat all kinds of pain caused by blood stasis [29]. “Materia Medica Huiyan”: “Safflower, broken blood also.”*Carthamus tinctorius* contains safflower glycoside and safflower quinone glycoside, which can dilate peripheral blood vessels, enhance fibrinolysis, reduce whole blood viscosity, effectively inhibit platelet aggregation, activate plasminogen, prolong clotting time, improve hemorheology, and improve hypoxia tolerance. Safflower yellow pigment has a strong and lasting analgesic effect, which is effective for both sharp pain and dull pain. Safflower preparation can inhibit the proliferation of vascular endothelial cells and has a significant effect on patients with diabetes mellitus complicated with peripheral atherosclerotic occlusive disease.

RETRACTED

Sappan wood: sweet and salty taste into the blood, with the effect of promoting blood circulation to treat injuries, relieving blood stasis, reducing swelling and relieving pain [27, 28]. It is a common medicine for gynecological stasis, menstruation, and other fatigue diseases. “New Materia Medica”: “the Lord breaks the blood, and the postpartum blood distension is boring to the dead.” “Rihuazi Materia Medica”: “treat women's blood gas, heart and abdominal pain, irregular menstruation and bed fatigue, discharge pus and relieve pain, reduce carbuncle swelling and blood stasis.” Sappan wood contains Brazilian hematoxylin, volatile oil, and tannin, which can promote microcirculation, inhibit platelet aggregation, and has antibacterial and anti-inflammatory effects. About 95% ethanol sappan wood extract has the effect of scavenging oxygen free radicals and superoxide anions, achieving antioxidation and protecting DNA damage induced by hydroxyl radicals. Some studies have indicated that sappan ethyl acetate and n-butanol can remarkably improve the incidence of insulitis in mice.

Jixueteng is good at enhancing blood circulation and tonifying blood, dispelling blood stasis, and reducing pain [28]. It is often adopted to treat menstrual disease of women with blood stasis and blood deficiency. This product tastes sweet, warm, bitter but not dry, warm but not strong, and gentle in nature and has the effect of relaxing muscles. It is often adopted to treat symptoms such as numbness and pain of hands and feet with obstruction of meridians and disharmony of collaterals. “decoction piece new ginseng”: “remove blood stasis, give birth to new blood, and fluent meridians.” “Compendium of Materia Medica”: “strong muscles and bones, soreness, and alcohol.” to treat the elderly, such as weakness of qi and blood, numbness of hands and feet, paralysis and so on.” It mainly contains isoflavones, triterpenes, and retention compounds, which have bidirectional regulation on the immune system, have obvious anti-inflammatory effects, and can also reduce vascular resistance. The total flavonoids of *Uncaria officinalis* can antagonize the antiplatelet aggregation induced by arachidonic acid. Other studies have indicated that soaking diabetic foot with papaya and *Tripterygium paniculata* decoction can dilate blood vessels and promote blood circulation of the foot. It can obviously improve the peripheral neuritis caused by CRI [29].

In conclusion, Mudan granule can remarkably facilitate the clinical symptoms of TCM and reduce the score of TCM syndrome in the treatment of peripheral neuritis caused by CRI; moreover, it can remarkably increase the nerve conduction velocity of median nerve and common peroneal nerve and reduce blood viscosity, which is worthy of clinical promotion.

RETRACTED

## Figures and Tables

**Figure 1:** Comparison of nerve conduction velocity between two groups of patients.

**Figure 2:** Comparison of hemorheological indexes between two groups of patients.

**Table 1:** Comparison of the curative effect [n%].

Group	*N*	Clinical recovery	Significant effect	Effective	Invalid	Total efficiency
C group	30	9 (30.00)	8 (26.67)	7 (23.33)	6 (20.00)	24 (80.00)
R group	30	22 (73.33)	5 (16.67)	3 (10.00)	1 (3.33)	29 (96.67)
*χ* ^2^						4.043
*P*						<0.05

**Table 2:** Comparison of TCM clinical symptom scores [$\bar{x}\pm \text{s}$, points].

Group	*N*	Limb numbness		Limb pain		Abnormal temperature sensation	
		Before treatment	After treatment	Before treatment	After treatment	Before treatment	After treatment
C group	30	4.82 ± 0.31	2.48 ± 0.55	4.13 ± 0.22	2.28 ± 0.35	3.84 ± 0.64	2.18 ± 0.21
R group	30	4.81 ± 0.22	1.35 ± 0.33	4.19 ± 0.25	1.66 ± 0.53	3.89 ± 0.68	1.39 ± 0.33
*t*		0.144	9.649	0.986	5.346	0.293	11.062
*P*		>0.05	<0.01	>0.05	<0.01	>0.05	<0.01

**Table 3:** Comparison of renal function indexes [$\bar{x}\pm \text{s}$].

Group	*N*	SCr (*μ*mol/L)		BUN (mmol/L)		UA (*μ*mol/L)	
		Before treatment	After treatment	Before treatment	After treatment	Before treatment	After treatment
C group	30	284.13 ± 33.21	241.95 ± 33.67	8.16 ± 1.24	8.03 ± 1.56	528.69 ± 22.54	481.95 ± 43.12
R group	30	285.18 ± 33.51	182.84 ± 33.22	8.19 ± 1.22	7.09 ± 1.04	528.91 ± 22.42	451.92 ± 42.31
*t*		0.121	6.844	0.094	2.746	0.037	2.722
*P*		>0.05	<0.01	>0.05	<0.01	>0.05	<0.01

**Table 4:** Comparison of inflammatory factor indexes before and after treatment [$\bar{x}\pm \text{s}$].

Group	*N*	IL-6 (pg/mL)		CRP (mg/L)	
		Before treatment	After treatment	Before treatment	After treatment
C group	30	41.83 ± 4.23	32.45 ± 2.46	67.94 ± 10.31	46.91 ± 3.31
R group	30	41.69 ± 4.45	26.39 ± 2.21	67.38 ± 10.34	39.49 ± 4.66
*t*		0.124	10.037	0.210	7.110
*P*		>0.05	<0.01	>0.05	<0.01

## Data Availability

The data was not available because of the patient information privacy.
